The article "Evaluation of the Risk of Recurrence in Patients with Local Advanced Rectal Tumours by Different Radiomic Analysis Approaches" was retracted in 2023. Reasons: signs of a paper mill; compromised peer review; unreliable results or conclusions.

# Evaluation of the Risk of Recurrence in Patients with Local Advanced Rectal Tumours by Different Radiomic Analysis Approaches

**DOI:** 10.1155/2021/4520450

**Published:** 2021-11-28

**Authors:** Alaa Khadidos, Adil Khadidos, Olfat M. Mirza, Tawfiq Hasanin, Wegayehu Enbeyle, Abdulsattar Abdullah Hamad

**Affiliations:** ^1^Department of Information Systems, Faculty of Computing and Information Technology, King Abdulaziz University, Jeddah, Saudi Arabia; ^2^Department of Information Technology, Faculty of Computing and Information Technology, King Abdulaziz University, Jeddah, Saudi Arabia; ^3^Department of Computer Science, College of Computers and Information Systems, Umm Al-Qura University, Makkah, Saudi Arabia; ^4^Department of Statistics, Mizan-Tepi University, Ethiopia; ^5^Tikrit University, College of Sciences, Iraq

## Abstract

The word radiomics, like all domains of type omics, assumes the existence of a large amount of data. Using artificial intelligence, in particular, different machine learning techniques, is a necessary step for better data exploitation. Classically, researchers in this field of radiomics have used conventional machine learning techniques (random forest, for example). More recently, deep learning, a subdomain of machine learning, has emerged. Its applications are increasing, and the results obtained so far have demonstrated their remarkable effectiveness. Several previous studies have explored the potential applications of radiomics in colorectal cancer. These potential applications can be grouped into several categories like evaluation of the reproducibility of texture data, prediction of response to treatment, prediction of the occurrence of metastases, and prediction of survival. Few studies, however, have explored the potential of radiomics in predicting recurrence-free survival. In this study, we evaluated and compared six conventional learning models and a deep learning model, based on MRI textural analysis of patients with locally advanced rectal tumours, correlated with the risk of recidivism; in traditional learning, we compared 2D image analysis models vs. 3D image analysis models, models based on a textural analysis of the tumour versus models taking into account the peritumoural environment in addition to the tumour itself. In deep learning, we built a 16-layer convolutional neural network model, driven by a 2D MRI image database comprising both the native images and the bounding box corresponding to each image.

## 1. Introduction

With advances in computer science and medical imaging, researchers have begun to explore new avenues for making the most of the information buried in medical images. Thus, radiomics emerged as a field of research in its own right and captured the attention of researchers. Radiomics is the extraction of a massive amount of data from conventional medical images, such as standard X-rays, ultrasound, CT scan, MRI, or even PET-scan, in correlation with the diagnosis, the stage of the disease, the therapeutic response, the genomic data, or relatively simple the prognosis [1]. It essentially emerged from cancerology, where providing specific information for personalized therapy is essential. Indeed, the same grade of the same histological type of a tumour can behave differently from one patient to another, hence the importance of personalized therapy [2]. The applications of radiomics in oncology are numerous. Rectal cancer is one of the most studied types of cancer by radiomic researchers. It is the third cancer in terms of morbidity and mortality [3]. Previous studies have reported that certain clinical-biological factors and conventional medical imaging may hold some predictive value, but a consensus has not been established [4, 5]. The role of radiomics as a potential predictive marker of recurrence has therefore been mentioned. Artificial intelligence and machine learning could help in the evaluation valuation of radiomic data. In particular, a deep understanding of convolutional neural networks (CNNs) could perform massive image texture analyses with minimal human input. However, there are limitations and challenges to overcome before radiomics can be implemented into routine clinical practice. Indeed, most radiomic studies conducted using conventional learning and published have been conducted with less than 100 patients [6]. We can see in deep learning an exciting alternative to traditional knowledge of machine techniques exploiting the potential of radiomics, in the sense that it allows the use of a small amount of raw data, few images, or patients, on which we could then apply an increase factor to increase the number of data without exposing the model to overlearning. At the same time, we will dispense with the manual segmentation of the tumour of interest, the manual extraction of radiomic data, and the problem associated with varying image preprocessing protocols. The present study evaluated and compared the predictive potential of conventional and deep learning algorithms applied to MRI scans of patients with locally advanced rectal tumours correlated with recurrence.

The article "Evaluation of the Risk of Recurrence in Patients with Local Advanced Rectal Tumours by Different Radiomic Analysis Approaches" was retracted in 2023. Reasons: signs of a paper mill; compromised peer review; unreliable results or conclusions.

## 2. Material and Methods

Indeed, most radiomic studies conducted using conventional learning and published have been conducted with less than 100 patients [7]. We can see in deep learning an exciting alternative to traditional learning of machine techniques exploiting the potential of radiomics, in the sense that it allows the use of a small amount of raw data, few images, or patients, on which we could then apply an increase factor to increase the number of data without exposing the model to overlearning. At the same time, we will dispense with the manual segmentation of the tumour of interest, the manual extraction of radiomic data, and the problem associated with varying image preprocessing protocols [7]. To test our hypothesis, we were faced with two issues:

- Were we going to use 2D or 3D images?
- Were we going to use only the tumour pixels, or would we include the peritumoural environment in a bounding box?

Initially, on conventional models, we tested the same database to predict recurrence, on 2D versus 3D algorithms, to show the noninferiority or even the superiority of the 2D models. Secondly, we tested the same database to predict recurrence on conventional models using masks from manual tumour segmentation versus bounding box masks to extract radiomic data. And lastly, we built the CNN model based on the results we got from testing conventional machine learning algorithms. In the rest of this report, we will present some generalities on radiomics and machine learning techniques, following the state of the art. We will detail the methodology used to carry out this study. Then, we will present the results obtained and discuss the essential data.

This component of the study, which was conducted as a distinct longitudinal research project, intended to elucidate further the relevance of the stable high-frequency characteristics found in the training sample in a different test dataset.

The feature extract was the same as the one described previously. We conducted comparisons at two different time points of cognitive stages to see if the levels in stable high-frequency characteristics were altered with cognitive decline. We used survival analyses to see if these features influenced the converting time of individuals.

## 3. Sample Selection

The present study comprises 98 patients, with an average age of 60 years, minimum of 21, maximum of 88 years, and male to female ratio of 2.065. Protocols varied depending on the machines used for image acquisition and among institutions. This variation was taken into account in the data analysis. Among the different MRI sequences available, the T2 sequence was chosen for the examination. This is for various reasons:

- Its informative character. Indeed, radiologists in their daily work rely on this type of footage for most of the interpretation
- Ubiquitous sequence. All MRI protocols included T2 lines
- Its particular interest in radiomics in rectal cancer which has already been demonstrated by numerous previous studies

For reasons of simplicity and computational difficulties, it was decided to ignore the other types of sequences.

The article "Evaluation of the Risk of Recurrence in Patients with Local Advanced Rectal Tumours by Different Radiomic Analysis Approaches" was retracted in 2023. Reasons: signs of a paper mill; compromised peer review; unreliable results or conclusions.

## 4. The Different Models Tested

- After manual segmentation, the conventional learning model, based on a 2D radiomic analysis of an image of interest from the MRI baseline (model 1)
- Conventional learning model, based on a 2D radiomic analysis of an MRI baseline bounding box (model 2)
- Conventional learning model, based on a 3D radiomic analysis of an image of interest from the MRI baseline, after manual segmentation (model 3)
- After manual segmentation, the conventional learning model, based on a 2D radiomic analysis of a post-MRI image of interest (model 4)
- Conventional learning model, based on a 2D radiomic analysis of an MRI post bounding box (model 5)
- After manual segmentation, the conventional learning model, based on a 3D radiomic analysis of a post-MRI image of interest (model 6)
- Deep learning model, based on a 2D analysis of the two MRI scans (baseline+posttherapy)

## 5. Raw Data

For each patient, a directory was created to organize the raw data. This directory contained six files:

- A DICOM file for T2 (3D) acquisition in the axial plane of the MRI baseline
- An NRRD file for 3D segmentation of tumour volume on MRI baseline
- An NRRD file for 2D segmentation of the tumour surface on MRI baseline. Segmentation was performed by choosing an image of interest from the acquisition volume image stack, ideally, the one passing through the epicentre of the tumour
- A DICOM file for T2 (3D) acquisition in the axial plane of the MRI post
- An NRRD file for 3D segmentation on the MRI post
- An NRRD file for 2D segmentation on the IRM post segmentation was performed by choosing an image of interest from the acquisition volume image stack, ideally, the one passing through the epicentre of the tumour. Reading the DICOM images and performing the segmentation were performed using free software, in everyday use: 3D Slicer, version 4.10.2

On baseline imaging, the volume or area of interest was defined by any wall thickening or mass syndrome appended to the rectal wall, appearing as an intermediate T2 signal, in diffusion restriction and enhanced after gadolinium injection. On posttreatment imaging, the volume or area of interest was defined by any morphological and signal abnormalities in place of the tumour being treated. The contouring of the lesions was performed by a radiologist manually, image by image for 3D segmentation and manually on a single image for 2D segmentation. Where there was any doubt about the pathological nature of the pixels, they were not taken into account in the segmentation. An Excel file was also created on which were noted the epicentres of the tumours (for the MRI baseline) and the epicentres of posttherapeutic changes (for the MRI post). Thus, after reading all the MRI scans, the *X*, *Y* and *Z* coordinates were collected on this file. These coordinates will be used for the creation of bounding boxes. The latter is created automatically for all patients on both the MRI baseline and the MRI post.  Figure 1 illustrates the three types of images used from an axial T2 sequence of the MRI baseline of the first patient of the training cohort.

The article "Evaluation of the Risk of Recurrence in Patients with Local Advanced Rectal Tumours by Different Radiomic Analysis Approaches" was retracted in 2023. Reasons: signs of a paper mill; compromised peer review; unreliable results or conclusions.

## 6. Conventional Learning Models

For each of these models, it has been implemented, the details of which can be found and the objectives of which are as follows:

- Automate the reading of raw images
- Automate the creation of bounding boxes
- Automate the preprocessing of images
- Automate the extraction of radiomic data
- Carry out the selection of informatic data
- Build a random forest model for binary classification
- The output of the model expressed as a binary variable (0 for no recurrence and 1 for recurrence)
- Train the model
- Test the performance of the model

### 6.1. Image Preprocessing

#### 6.1.1. A Resampling Step

Due to variation in protocols and the inhomogeneity in pixel size between different patients and different images, Figure 1 shows that this step was necessary. Before resampling, the pixel size was between 0.5 and 0.9 in the *X* and *Y* dimensions and between 2.5 and 4 in the *Z* dimension. The resampling used a function available on the radiomics library, with as output images of pixels with 1 × 1 mm in the *XY* plane and 4 mm in *z* depth. A normalization step used the “normalize” function of radiomics. As a reminder, normalization is a process of changing the intensity dynamics of the pixels so that the samples are comparable. In our case, the dynamics of the intensities of the pixels was fixed on an interval of 0 to 255. In addition to the original image, several filters have been applied to increase the amount of data extracted and make the most of the information in the picture.

A total of 8 filters were applied: Wavelet, LoG (Laplacian of Gaussian), Square, Square Root, Logarithm, Exponential, Gradient, and LBP2D or LBP3D.

- The Wavelet filter returns several decompositions (all combinations are possible by applying a high-pass or low-pass filter, the interest being to remove noise)
- The Laplacian of Gaussian filter will be used for contour enhancement, identifying areas of change in intensity
- The Square filter squares the intensities of the pixels
- The Square Root takes the square root of the intensities of the pixels
- The Logarithm filter takes the logarithm of the intensities of the pixels
- The Exponential filter, as its name suggests here again, exponentially puts the intensities of the pixels
- The Gradient filter returns the magnitude of the gradient
- The LBP2D filter returns a local binary pattern in 2D
- The LBP3D filter returns a local binary pattern in 3D using spherical harmonics. The last image returned corresponds to the kurtosis map

The article "Evaluation of the Risk of Recurrence in Patients with Local Advanced Rectal Tumours by Different Radiomic Analysis Approaches" was retracted in 2023. Reasons: signs of a paper mill; compromised peer review; unreliable results or conclusions.

### 6.2. Extraction of Radiomic Data

The data was extracted, in an automated way using the algorithm implemented, from the original image and the images built by applying the eight filters previously mentioned. The extraction process was performed for each model, with over 1000 radiomic data recovered/patient.

The whole thing was organized in a data frame on it.

### 6.3. Data Selection

The question of selecting data or attributes for classification is a very active line of research in data mining. This selection makes it possible to identify and eliminate the variables that penalize the performance of a complex model insofar as they may be noisy, uninformative, redundant, or not (or not very) reproducible. In addition, the identification of relevant variables considerably facilitates the interpretation and understanding of the radiological aspects of tumours. It also improves the prediction performance of the classification algorithm and overcomes the curse of dimensionality. In our study, the number of variables was much greater than the number of patients or observations (a factor of 10-15), making “selection” necessary. The machine learning literature has described three approaches: the filter, wrapper, and embedded approach. As shown in Figure 2, the latter two implicitly select variables during the learning process, unlike the first. The first is to go through all of the data before the learning process.

In this context, we opted for a combinatorial technique, Figure 2, using both a selection algorithm (recursive feature elimination or RFE) with a classification algorithm (random forest or RF). This approach is relatively easy to implement and has already been shown to be effective. RFE is a technique that selects predictive data retrograde. She starts by building the RF model, using all the radiomic data available in the training game. It calculates a critical factor for each data. The data with the lowest importance factors is discarded with each iteration. A parameter is used to adjust the number of variables eliminated on each iteration. In our study, it was set at 50. A recalculation of the critical factors for the remaining data is performed during the next iteration until the most predictive data is obtained. RF is often used with RFE because it does not exclude variables from the prediction equation and because RF has a well-known internal method for calculating the importance of data. The other advantage of this technique is that the optimal number of data to be selected for constructing the predictive model is automatically given at the end of the analysis.

The article "Evaluation of the Risk of Recurrence in Patients with Local Advanced Rectal Tumours by Different Radiomic Analysis Approaches" was retracted in 2023. Reasons: signs of a paper mill; compromised peer review; unreliable results or conclusions.

### 6.4. Construction of the Model

The construction of the predictive model used the “random forest” algorithm (or RF for random forest). It is an algorithm combining many decision trees in a bagging-type approach. According to resampling techniques, bagging or bootstrap is a group of statistical inference methods based on the multiple replications of the studied dataset. Thus, each decision tree receives part of the initial dataset. A decision tree [8] is a graphical visualization of a series of decisions/possibilities in the form of a tree. Each point is a node, and each link between nodes is a branch. The starting point is at the top of the tree, and the decision/final state is at the other end: this is reached by following a path defined by the intermediate steps at each node separated into two subgroups. The RF assigns a probability to each path/exit point combination. The best-known segmentation criterion for the classification problem is the Gini impurity index. The concept of purity refers to the discriminating nature of the separation effected by a node.

### 6.5. Performance Analysis

For each model trained, we performed an iteration to acquire the confusion matrix and calculate a precision factor on a test cohort representing 50% of the initial dataset.

### 6.6. Performance Comparison

This was done by comparing the resulting 5 AUC values for each of the six models. Considering the nonnormal distribution and the comparison of different groups of values (>2), a nonparametric test such as Kruskal-Wallis was necessary. The alpha risk threshold for concluding a difference was set at 0.05.

## 7. Deep Learning Model

### 7.1. Data Organization

To build a powerful and efficient neural network, an extensive database was necessary. To do this, we grouped all the images in a single database, namely, the 98 pictures of the MRI baseline ×2 (raw and bounding box) and the 98 photos of the MRI post ×2 (natural and bounding box). In total, we had 392 images. Patients were randomized into training and validation cohorts at a ratio of 0.8. The images were resampled to have dimensions of 224 × 224 to avoid changing the basic architecture of the neural network.

### 7.2. Data Augmentation

To take full advantage of the potential of the neural network, we have added a data augmentation factor. Kora's library contained functions capable of handling the initial images and performing some modifications to build images with different information.

The article "Evaluation of the Risk of Recurrence in Patients with Local Advanced Rectal Tumours by Different Radiomic Analysis Approaches" was retracted in 2023. Reasons: signs of a paper mill; compromised peer review; unreliable results or conclusions.

This increase in data called on

- randomization for each of the data (this being obtained by dividing the value by the average of all the values)
- random rotations in an interval of 20°
- displacements in the *x* and *y* axes over lengths corresponding to 0.2 of the matrix dimension
- last to horizontal flips

## 8. Results and Discussion

### 8.1. Description of the Study Population

The present study comprises a total of 98 patients. With an average age 60 years, minimum 21, maximum 88 years, and male to female ratio 2.065, given the imbalance between the number of patients having recurrence (24/98) and the number of patients without recurrence (64/98), a sampling technique increasing the size of the minority sample was necessary to have the same number of observations per sample. For this, we applied SMOTE (for the acronym synthetic minority oversampling technique).

### 8.2. Performance of Conventional Learning Models

The summary of performance results for each model is shown in Table 1.

**Model 1 .**

1045 radiomic data were extracted for each patient.

After applying the selection algorithm, 28 data items were saved as the radiomic signature.

1-Display Script. Results of the radiomic data selection for model 1

('Optimal number of features:' 28)

('Best features:' Index ([33, 40, 45, 52, 67, 71, 76, 86, 98, 106, 114, 120, 125, 149, 151, 186, 205, 254, 279, 355, 935, 959, 963, 964, 979, 991, 1026, 1041],

dtype='object')]

The result of testing the model's performance on the validation cohort is shown:

- On an iteration in the form of a confusion matrix

Note that on this confusion matrix, the performance was more significant than 0.9

(ii) On all the cross-validation iterations in the form of ROC curves (receiver operating characteristic) (not given here)

Note in particular an area under the average curve estimated at 0.83 ± 0.08

2-Display Script. Confusion matrix for model 1

= = = Confusion Matric = = =

[[36 6]

[0 32]]

On this confusion matrix, on the first column, we find the number of patients without recurrence, on the second column the number of patients with recurrence, on the first line the number of patients labelled by the model as being at low risk of recurrence, and on the second line the number of patients labelled by the model as being at high risk of recurrence.

**Model 2 .**

1046 radiomic data were extracted for each patient.

After applying the selection algorithm, 22 data items were saved as the radiomic signature.

Results of radiomic data selection for model 2.

The article "Evaluation of the Risk of Recurrence in Patients with Local Advanced Rectal Tumours by Different Radiomic Analysis Approaches" was retracted in 2023. Reasons: signs of a paper mill; compromised peer review; unreliable results or conclusions.

The result of testing the model's performance on the validation cohort is shown:

('Optimal number of features:' 22)

('Best features:' Index ([31, 35, 36, 41, 45, 47, 48, 56, 61, 76, 80, 102, 110, 112, 114, 135, 212, 253, 776, 984, 991],

dtype='object')]

- On an iteration in the form of a confusion matrix.

Note that on this confusion matrix, the performance was greater than 0.65

(ii) On all the iterations of the cross-validation in the form of ROC curves. Note in particular an area under the average curve estimated at 0.80 ± 0.12

Confusion matrix for model 2 ROC curves for model 2.

= = = Confusion Matric = = =

[[27 12]

[14 21] ]

## 9. Performance Comparison of Conventional Learning Models

The performance in terms of AUC was compared between the six models using the Kruskal-Wallis test. The result is shown in the screenshot below.

The results in fact show that there is no difference between the performances of the 6 models.

Script. Performance comparison of the 6 conventional learning models

(1)from scipy.stats import kruskal

(2)X6 = [0.63, 0.67, 0.77, 0.87, 0.89]

(3)X5 = [0.75, 0.83, 0.87, 0.83, 0.87]

(4)X4 = [0.86, 0.9, 0.8, 0.8, 0.67]

(5)X3 = [0.68, 0.9, 0.67, 0.73, 0.8]

(6)X2 = [0.89, 0.73, 0.7, 1, 0.7]

(7)X1 = (0.75, 0.93, 0.9, 0.83, 0.73]

(8)stat, p = kruskal (X1, X2, X3, X4, X5, X6)

(9)print (‘Statistics = %.3f, p = %.3f′%(stat, p))

(10)# interpret

(11)alpha = 0.05

(12)if p > alpha:

(13)-----_∗_print("Same distributions (fail to reject H0)')

(14)else:

(15)-----_∗_print("Different distributions (reject H0)')

Statistics-2.675, p = 0.750

Identical distributions (fail to reject H0)

The trainable dataset was calculated as 134,268,738.

In Table 2 the learning phase, our model has not shown itself capable of learning. After 25 epochs, the model showed performances close to 0.5 (by chance), with nonconvergent loss functions and a single-class prediction.

## 10. Discussion

### 10.1. Conventional Learning

- *Performance of Each Model*. The results of conventional learning models agree with what has been published previously. Indeed, the six models showed a specific predictive capacity, with *p* values remaining below the alpha threshold of 0.05, once again underlining the potential of radiomics as a predictive factor, in particular of the risk of recurrence of locally advanced rectal neoplasias and its interest in the selection of high-risk patients
- *Comparison of Model Performance*. In our study, the Kruskal-Wallis test highlights two main results:
- The lack of significant difference between models using 2D data vs. models using 3D data
- The noninferiority of models using the bounding box compared to models using tumour contouring

What more do we bring to literature? Their study evaluating 2D vs. 3D data used CT images on lung sections [9–13]. However, we know that what applies to a given imaging modality (CT, MRI, ultrasound, etc.) does not necessarily apply to another modality. In addition, anatomy is a factor to consider. The scanner is suitable for analyzing the lung parenchyma, and it is terrible for the local evaluation of rectal cancer.

The article "Evaluation of the Risk of Recurrence in Patients with Local Advanced Rectal Tumours by Different Radiomic Analysis Approaches" was retracted in 2023. Reasons: signs of a paper mill; compromised peer review; unreliable results or conclusions.

Conversely, MRI is very efficient for evaluating rectal cancer, with minimal indications in evaluating bronchopulmonary cancer. To our knowledge, no previous study has assessed the performance of 2D vs. 3D texture data on MRI images. The advantage of 2D data is undeniable in terms of calculation time and simplicity of the models. The results of our study, therefore, support the use of 2D data.

The performance of models using the bounding box remains comparable to other conventional learning models. Although not inferior, it was not superior in terms of prediction within sample size limits. This bounding box role has already been evoked by Hosni A and Al. who has suggested the presence of information at the level of the immediate peritumoural environment [13–22]. Although in our study we failed to demonstrate the existence of predictive information within this immediate environment, this idea of bounding box is not obsolete because it limits human input. In other words, the radiologist does not have to segment the tumour but clicks on the epicentre of the tumour and retrieves the *x*, *y*, and *z* coordinates of that epicentre which are done automatically. We will add pixels on either side of these coordinates according to a number that we define.

## 11. Problem of Deep Learning

Our CNN model did not show any predictive potential.

To understand this result as well as possible, we first checked the outputs of the model. These were all of the same class: either it is 0 or it is 1. Secondly, we sought to understand the reasons behind this neural network giving as outputs a unique style. A small tour of the literature allows us to collect some hypotheses concerning this problem:

- Error related to the type of pixel values
- The architecture of the neural network itself
- Learning misses too high or too low
- Image preprocessing
- “A dying ReLU”
- A neural network that is too deep
- Finally, the lack of correlation between entry (MRI images) and prognosis

- It is claimed that there is no error related to the type of pixel values. These have been verified several times. The values were expressed in float64
- We do not think the error is related to the architecture of the network. We tried several experiments with the addition and removal of different layers
- Concerning the learning rate, again, several experiments were tested with values between 0.001 and 0.5. The problem persists with all of the values tested
- According to the state-of-the-art data, the preprocessing of the images has been correctly carried out
- The concept of dying ReLU refers to the fragility of the ReLU activation function. When a large gradient passes through the ReLU neuron, it may change the weights so that this neuron will not activate during subsequent iterations. The result is that the dead ReLU neuron will always give the same output. To overcome this problem, one tested instead of the ReLU functions the “leaky ReLU” function. According to the following formula, this was supposed to give a slight positive gradient when the input was negative (*y* = 0.03*x* when *x* < 0, with *x* as input and *y* as output). This leaky ReLU function was supposed to solve the problem of neuronal death, but the model remains in single-class prediction, even after changing the activation functions
- The network depth does not seem to be a problem since different depths have been tested, from the 11-layer model to the 19-layer model
- Conventional machine learning models were able to capture the predictive information buried in the MRI images of our database in correlation to the risk of recurrence. Therefore, we reject the hypothesis that the failure of the deep learning model can be justified by the lack of correlation between the data and the prognosis

Therefore, it turns out that convolutional neural networks process information from MRI images entirely differently than conventional learning techniques. Where traditional methods receive texture data as input resulting from a straightforward and relatively easy form of engineering, the texture analysis performed in the dark by CNNs which appears different and challenging to understand. Thus, CNNs are not to date an automatic equivalent to conventional learning techniques, contrary to what was assumed at the start of the study. Although they have the advantage of certain automaticity and simplicity of execution, they deserve their “black box” qualifier.

The article "Evaluation of the Risk of Recurrence in Patients with Local Advanced Rectal Tumours by Different Radiomic Analysis Approaches" was retracted in 2023. Reasons: signs of a paper mill; compromised peer review; unreliable results or conclusions.

## 12. Conclusion

This study evaluated and compared six conventional learning models and one deep learning model, based on MRI textural analysis of patients with locally advanced rectal tumours, correlated with the risk of recurrence. In conventional learning, we compared 2D image analysis models vs. 3D image analysis models, models based on a textural analysis of the tumour versus models taking into account the peritumoural environment in more of the tumour itself. We built a 16-layer convolutional neural network model in deep learning, driven by a 2D MRI image database comprising both the native images and the bounding box corresponding to each image. Conventional education is highly effective, with each model having radiomic signatures capable of accurately predicting the risk of recurrence. Conversely, deep learning was unable to learn patterns correlated with prognosis. It does not constitute an automatic substitute for more conventional techniques, contrary to what has been suggested. Comparing the performance of traditional learning models with each other highlights two main facts. First, where 3D texture data has the disadvantage of being complex and requiring time and significant computational capacity, 2D texture data has shown equivalent performance with the advantage of simplicity and lower cost in computing skills. Second, at the risk of being time-consuming, the manual segmentation before the extraction of texture data in conventional learning can be replaced by the quasiautomatic creation of bounding boxes, less costly in time and energy, and including a peritumoural environment potentially valuable for the performance of the model.

## Figures and Tables

**Figure 1:** Example illustrating the 2D segmentation and the bounding box with the corresponding native image on an MRI baseline native image on the left, 2D segmentation in the middle, and bounding box on the right.

**Figure 2:** Data selection by the wrapper and embedded approach.

**Code 1:** Network training result

**Code 2:** Model predictions on the validation cohort

**Table 1:** Summary results of conventional learning model performance.

Templates	Number of radiomic data extracted	Number of data selected and included in the radiomic signature	The precision of the model on the confusion matrix	AUC average over the five iterations	*p* value
1	1045	28	0.91	0.83 ± 0.08	0.001
2	1046	22	0.68	0.8 ± 0.12	0.001
3	1632	8	0.65	0.76 ± 0.09	0.001
4	1045	21	0.73	0.8 ± 0.08	0.001
5	1046	22	0.81	0.83 ± 0.04	0.001
6	1632	8	0.74	0.83 ± 0.08	0.001

**Table 2:** Number of parameters that the network can train.

Wax pooling24 15 (MaxPooling)	(None, 7, 7, 512)	0
Flatten_3 (flatten)	(None, 25088)	0
dense_7 (dense)	(None, 4096)	102764544
dropout 8 (dropout)	(None, 4096)	0
dense_8 (dense)	(None, 4096)	16781312
dropout (dropout)	(None, 4096)	0
dense_9 (dense)	(None, 2)	8194
=========================================================================		
parama: 134,268,738		
Trainable parans: 134,268,738		
Nontrainable params: 0		

## Data Availability

The data used to support the findings of this study are included within the article.
